# Design and Clinical Application Effect Analysis of a New Type of Oral Fluid Suction Device for Patients with Orotracheal Intubation

**DOI:** 10.1155/2022/6057115

**Published:** 2022-07-20

**Authors:** Yanying Qian, Haifei Lu

**Affiliations:** Surgical Intensive Care Unit, The Second Affiliated Hospital of Zhejiang University, Hangzhou, Zhejiang 310009, China

## Abstract

Tracheal intubation is an important access to general anesthesia surgery or respiratory support in critically ill patients. Orotracheal intubation is the most common method of establishing artificial airways in clinical practice. Tracheal intubation and mechanically assisted breathing are among the important steps in the clinical rescue of critically ill patients. During tracheal intubation, it easily causes iatrogenic skin damage, unclear mouth, ulcer, and other oral mucosal complications due to the improper fixation method and excellent dental pads. Therefore, the purpose of this study was to design a novel oral suction device for patients with orotracheal intubation and explore its safety, convenience, and comfort in the clinical application of orotracheal intubation patients. From October 2016 to April 2017, a total of 232 patients with mechanical ventilation through orotracheal intubation in the Department of Surgery and Critical Care Medicine were selected by the convenience sampling method. According to the random number table method, 232 cases were divided into the experimental group and control group, with 116 cases in each group. The experimental group used a self-designed oral fluid suction device to fix the tracheal intubation; the control group used the traditional method, placing ordinary disposable tooth pads, and then using 3M tape to fix the tracheal intubation. The incidence of oral mucosa and lip pressure ulcers, patient comfort, and tracheal tube displacement were observed and compared between the two groups. The incidence of oral mucosa and lip pressure ulcers in the observation group using the self-designed oral fluid suction device to fix the tracheal intubation was significantly lower than that in the control group. At the same time, the comfort of the patients was significantly higher than that of the control group, the incidence of tracheal tube displacement was significantly lower than that of the control group, and the differences between the above indicators were statistically significant (*P* < 0.05). For patients with orotracheal intubation, using a new oral fluid suction device to fix the tracheal intubation can effectively prevent the displacement of the tracheal intubation, protect the oral mucosa and lips, and reduce the pain of the patient. At the same time, the oral fluid suction device designed in this study has low production cost, strong practicability, and is suitable for clinical promotion.

## 1. Introduction

Tracheal intubation is an important channel for breathing support for patients undergoing general anesthesia surgery or critically ill patients. Orotracheal intubation is the most commonly used method for establishing artificial airways in clinical practice. Tracheal intubation and mechanically assisted breathing are one of the important steps in the clinical rescue of critically ill patients [1]. During orotracheal intubation, due to improper fixation methods and excellent dental pads, it is easy to cause iatrogenic skin damage, oral uncleanness, ulcers, and other oral mucosal complications. The appearance of these problems not only causes discomfort to patients and increases pain but also increases the workload of nursing staff and affects work efficiency. Some studies [2, 3] have pointed out that no matter which medical operation the dental pads are used for, there will be a problem that is easily overlooked by medical staff, that is, pressure ulcers on the lips. Occurrence of lip pressure ulcers increases pain for intubated patients [4]. The presence of the tooth pad will occupy a certain space in the oral cavity, so that the patient passively opens the mouth. This passive mouth opening stimulates the increase of oral secretions. If the oral secretions are not sucked out in time, the stability of the tape for fixing the endotracheal intubation device will be affected, and the risk of unplanned extubation will be increased. Timely replacement and regular suction removal of patient oral secretions greatly increase the workload of nursing staff. Aiming at the problems of oral pressure ulcers and frequent removal of oral secretions caused by orotracheal intubation, this study designed a new oral fluid suction device for patients with orotracheal intubation and applied this device to the clinic. At the same time of removing oral secretions, it can prevent the displacement of tracheal intubation, protect the oral mucosa and lips, and improve the comfort of patients.

## 2. Materials and Methods

### 2.1. Research Methods

232 patients with mechanical ventilation through orotracheal intubation in the Department of Surgery and Critical Care Medicine from October 2016 to April 2017 were chosen as the research subjects. Inclusion criteria were as follows: age ≥ 18 years old; first intubation after admission; all patients underwent orotracheal intubation for mechanical ventilation; no coagulation dysfunction; no patients with pulmonary infection; no oral disease; days of orotracheal intubation ≥ 2 days; tracheal intubation; and the skin around the mouth, cheeks, and neck before the tube was intact without ulceration. Exclusion criteria were as follows: patients with severe oral diseases; patients with severe bleeding and coagulation disorders; oral infection; those with respiratory tract infection and pulmonary infection before tracheal intubation; those who do not actively cooperate with the researcher; and those with mental illness and communication disorders. The investigation of this study was carried out with the consent of nurses and patients and signed a voluntary informed consent form. The study protocol has been reviewed and approved by the hospital ethics committee. According to the random number table method, 232 patients were divided into the experimental group and the control group, with 116 cases in each group. General information is given in Table 1. There was no statistical difference in age, gender, and disease composition between the experimental group and the control group (*P* > 0.05), and the two groups of patients were comparable.

### 2.2. Research Method

#### 2.2.1. Design and Manufacture of Oral Fluid Suction Device

The oral liquid suction device includes a guide tube and a liquid suction body. The side wall of the top is inwardly recessed to form a circular groove. The liquid suction body is cylindrical, and its diameter gradually decreases from the top to the bottom. The main body is used to absorb oral fluid, which is made of multiple layers of gauze wound in a spiral manner. The adjacent gauze layers of each layer are stacked in sequence. The liquid absorbing body includes a first body, a second body, a third body, and a fourth body. They are sequentially stacked from the inner ring to the outer ring. The liquid body is formed by winding a piece of gauze with flushing seam covered by adjacent layers of gauze. One end of the guide tube is inserted into the suction body from the top of the suction body; the other one is exposed to the suction body. One that is exposed to the suction body is used for connecting with the negative pressure suction device. The side wall of the guide tube inserted in the suction body has several guide holes. While oral liquid in the suction body flows into the guide tube through the guide holes, the suction body is passed through the guide tube and the oral fluid in the duct is discharged. The diversion tube includes a first diversion tube and a second diversion tube. One end of the first diversion tube is connected with one end of the second diversion tube. The first diversion tube is located in the suction body inside and the second is located outside. The outer wall of the end connected with the second guide tube is recessed inward to form a ring-shaped slot, and the second guide tube is connected to the second guide tube. The inner wall of the connected end of a guide tube protrudes to form a ring-shaped clamping table, and the ring-shaped clamping table is clamped into the circular clamping groove and can rotate in the circular clamping groove. A sealing ring is installed between the ring-shaped clamping table and the ring-shaped clamping groove. Production materials are as follows: 4 pieces of self-sealing gauze 8 cm ∗ 30 cm, 1 piece of 4 mm (12F)  ∗ 550 mm suction tube, 1 piece of 3M sterilized breathable film 6 cm ∗ 7 cm, and a pair of scissors. Made according to the method above, the product is a one-time use, as shown in Figure 1.

#### 2.2.2. Intervention Method

When the patients have been successfully intubated by the orotracheal tube, the control group placed ordinary disposable dental pads between the upper and lower teeth of patients. The experimental group used an oral fluid suction device (Has obtained the utility model patent of the State Intellectual Property Office of the People's Republic of China, Number of the patent: ZL 2016 20533942.0). Placed between the upper and lower teeth, the dental pad and the tracheal tube were tied side by side with tape and then fixed on the patient's cheeks with 3M tape [5]. After successful tracheal intubation in both groups, the exposed length of the tracheal cannula was determined, surrounded the tracheal tube by an ordinary tape of about 2 cm and marked cautiously to value the displacement of it [6].

### 2.3. Objective Indicators and Evaluation Criteria

#### 2.3.1. The Incidence of Oral Pressure Ulcers in the Two Groups of Patients during Mechanical Ventilation through Orotracheal Intubation Was Compared

The occurrence of pressure sores on the lips was evaluated before each oral care. According to the staging of oral ulcers, stage 1 pressure ulcers: flaky or streak-like bruising on the skin around the lips and gums; stage II pressure ulcers: the skin around the lips and gums is purple-red, with blisters and superficial mucosal ulceration; and stage III pressure ulcer: A superficial ulcer stage, with full-thickness skin destruction, which can penetrate deep into the subcutaneous tissue and deep tissue [7].

#### 2.3.2. Patient Comfort Assessment

Patients were assessed by uniformly trained nurses. According to the patient's self-perception, a visual analog scale (VAS) was used, with 0 indicating comfort, 5 indicating general comfort, and 10 indicating very uncomfortable. Higher scores indicate lower comfort levels.

#### 2.3.3. The Degree of Displacement of Tracheal Intubation [8]

(1) No displacement: the graduation of the catheter tip from the incisors was completely unchanged. (2) Mild displacement: the distance between the tip of the catheter and the scale of the incisor teeth is within 0.5 cm. (3) Moderate displacement: the distance between the tip of the catheter and the scale of the incisors is 0.5–0.8 cm up and down, but it does not cause the catheter to fall off or slide down to one main bronchus. (4) Severe displacement: the tube is dislodged or the tube slides down and blocks one side bronchus.

### 2.4. Statistic Method

SPSS 19.0 was used to analyze the data, the quantitative materials fit a normal distribution. The quantitative data are presented by (*χ* ± SD). Comparisons of materials between two groups were performed by the *t*-test. The enumeration data were expressed as percentages, the comparison of the enumeration data was performed by the chi-square test, and the comparison of the rank data between groups was performed by the Wilcoxon rank-sum test. Differences between groups were considered statistically significant at *P* < 0.05.

## 3. Results

### 3.1. Comparison of Oral Mucosa and Lip Pressure Ulcers between Two Groups of Patients

There were no severe oral mucosal and oral pressure ulcers in both groups. The incidence of oral mucosa and lip pressure ulcers in the observation group after intubation was significantly lower than that in the control group, and the difference was statistically significant (*P* < 0.05), as given in Table 2.

### 3.2. Comparison of Changes in Comfort of Two Groups of Patients

The comfort of the patients in the experimental group after intubation was significantly better than that in the control group, and the difference was statistically significant (*χ*^2^ = 30.034, *P* ≤ 0.001), as given in Table 3.

### 3.3. Comparison of Tracheal Tube Displacement in Two Groups of Patients

Severe displacement did not happen in both groups of patients. The degree of displacement in the experimental group is significantly smaller than in the control group. The difference was statistically significant (*P* < 0.05), as given in Table 4.

## 4. Discussion

Tracheal intubation is the most basic rescue technique for critically ill patients. It is of great significance in the maintenance of airway patency, ventilation and oxygen supply, airway suction, and prevention of aspiration [9]. Orotracheal intubation is widely used in clinical practice, but it is prone to the shortcomings of accidental extubation, oral complications, and incomplete oral evaluation [10], which lead to the occurrence of doctor-patient disputes. With the innovation of nursing technology, the fixation materials and methods of orotracheal intubation are constantly updated. While paying attention to the fixation effect, nurses also pay attention to improving the comfort of patients and choose personalized and appropriate fixation methods for different patients [11]. The traditional fixation method is fixed with silk tape. After fixation, the silk tape is easily curled and loosened after being contaminated by the patient's secretions, vomitus, and sweat, resulting in the risk of displacement or prolapse. It needs to be replaced and fixed again. Low sex [12] increases the workload of nurses. The traditional method of fixing the tracheal intubation makes the patient's mouth in a closed state. Oral care needs to be removed after the adhesive tape and tooth pads are removed. After oral care, the tracheal intubation should be refixed. Repeated replacement of the silk tape or daily oral care often requires 2 people. It can only be completed with assistance, which also increases the nursing time and cost. In busy work, it will affect the quality of patients' oral care. In this study, by designing a new oral fluid suction device for patients with orotracheal intubation and applying it to clinical work, it was found that it has many significant advantages.

In actual work, the material of ordinary disposable dental pads is hard, and its flanks are easy to compress the skin of the patient's lips, resulting in damage to the skin there. For patients with missing dentition, the dental pad is in direct contact with the gums, and prolonged pressure will damage the gums. In addition, the back of the tooth pad is narrow, and there is general physical friction between the lingual surface and the upper jaw. These physical frictions can easily lead to damage to the oral mucosa and easily lead to oral complications. The oral liquid suction device designed in this study has a cylindrical body with no side wings, which reduces the friction between the device and the lips, oral mucosa, teeth, and gums. At the same time, the material of the device is gauze, which acts as a buffer between the tooth pad and the gums for patients with missing dentition, which greatly reduces the hardness and reduces pressure on the teeth and gums.

In the traditional method, the common dental pads are mostly straight-shaped wings, which are made of a very hard plastic product, which is easy to compress the lips and gums, causing discomfort. The main material of the newly designed oral fluid suction device in this study is gauze, which changes the original plastic shell structure column, avoids pressure on the perioral skin, and improves the comfort of the patient. In traditional operations, nurses need to use a suction tube to suck the secretions in the mouth of patients with endotracheal intubation through the tooth pad. Such manipulation can stimulate nausea and even vomiting in the patient. After adopting the newly designed oral liquid suction device, the end of the guide tube is directly connected with the negative pressure suction device, which reduces the stimulation of the patient's oropharynx and increases the patient's comfort.

In critically ill patients in the intensive care unit, due to endotracheal intubation and matching tooth pads, the patient's mouth cannot be closed voluntarily, and the swallowing function is limited. This situation can easily lead to difficulties in excretion of oral secretions and changes in saliva properties. Furthermore, under the influence of various factors, the oral environment of patients may even be disturbed, bacterial reproduction will increase, and oral cleanliness will be significantly reduced [13]. The average daily oral secretion of fluid is 500–1500 ml. After intubation, due to the stimulation of the material, the oral secretion of liquid continues to increase, resulting in the infiltration of the tape, which affects the stable function of the tape. This greatly increases the risk of displacement of the endotracheal tube. A study [14] pointed out that one case of unplanned extubation was precise because the patient's oral secretions soaked the fixation tape. At the same time, the nurse did not change the tape in time, causing the patient to push out the tooth pad with his tongue and take out the tracheal intubation. Unplanned extubation is a serious complication of endotracheal intubation. Foreign studies have shown that the incidence of unplanned extubation of endotracheal intubation is 3%–16% [15], and domestic reports are 5.4%–15.5% [16]. The end of the guide tube of the oral liquid suction device is connected with the negative pressure suction device, which can suck out the oral liquid in time, avoid gauze infiltration due to excessive oral liquid, and greatly reduce the risk of displacement of the tracheal intubation. There is a ring-shaped groove at the top of the suction device body, and the patient's teeth or gums directly contact here, which ensures the stability of the catheter and will not move at will.

## 5. Conclusion

The oral fluid suction device provided by the utility model has the advantages of simple structure and convenient use, which solves the problem that the oral fluid of the patient cannot be easily sucked out and increases the operation difficulty of the medical staff. The oral fluid suction device can not only quickly suck out the oral fluid and avoid pressure sores on the patient's lips and damage to the oral mucosa but also ensure the comfort of the patient, and at the same time, it is convenient for medical staff to use the oral fluid suction device, and the work efficiency is improved. In addition, the oral liquid suction device has low manufacturing cost, strong practicability, and is suitable for promotion.

## Figures and Tables

**Figure 1:** Design drawing of the oral fluid suction device.

**Table 1:** General data of patients in the experimental group and control group.

Grouping	The number of cases	Gender (example %)		Age (years)	The cause of surgery
		Male	Female		
The experimental group	116	80 (68.97)	36 (31.03)	63.25 ± 2.6	116
The control group	116	72 (62.07)	44 (37.93)	61.81 ± 3.4	116

**Table 2:** Comparison of oral and lip pressure sores and labial pressure ulcers between two groups (case).

Group	The number of cases	Oral and lip pressure				Oral cavity mucous membrane	
		Without	Mild	Moderate	Severe	Exist	Without
The experimental group	116	115	1	0	0	1	115
The control group	116	100	14	2	0	10	106
*χ* ^2^ values			12.297	2.276		4.683	
*P* values			*P* < 0.0001	*P*=0.131		*P* < 0.05	

**Table 3:** Changes in the comfort level of patients in two groups (case).

Group	The number of cases	Comfortable	General	Not comfortable
The experimental group	116	100	15	1
The control group	116	50	45	21
*χ* ^2^ values			30.034	20.087
*P* values			*P* < 0.0001	*P* < 0.0001

**Table 4:** Comparison of displacement degree of the tracheal tube between two groups (case).

Group	The number of cases	Without	Mild	Moderate	Severe
The experimental group	116	114	1	0	0
The control group	116	110	14	2	0
*χ* ^2^ values			12.297		
*P* values			*P* < 0.0001		

## Data Availability

The data used to support the findings of this study are available from the corresponding author upon request.
